# Interferon-*γ* Stimulates Interleukin-27 Derived from Dendritic Cells to Regulate Th9 Differentiation through STAT1/3 Pathway

**DOI:** 10.1155/2022/1542112

**Published:** 2022-10-18

**Authors:** Peng Xiong, Tonglin Liu, Yu Chen, Qianqian Xu, Xiaolin Hu, Fei Han, Lili Shi

**Affiliations:** ^1^Department of Pediatrics, Tongji Hospital, Tongji Medical College, Huazhong University of Science and Technology, Wuhan 430030, China; ^2^Department of Gastrointestinal Surgery, Union Hospital, Tongji Medical College, Huazhong University of Science and Technology, Wuhan 430030, China; ^3^Department of Otolaryngology-Head and Neck Surgery, Tongji Hospital, Tongji Medical College, Huazhong University of Science and Technology, Wuhan 430030, China

## Abstract

The initiation and progression of allergic asthma (AA) are associated with complex interactions between inflammation and immune response. Herein, we report the specific mechanisms underlying the molecular action of interferon (IFN)-*γ* in AA regulation. We speculated that IFN-*γ* inhibits Th9 differentiation by regulating the secretion of interleukin (IL)-27 from dendritic cells (DCs), thereby suppressing airway inflammation in asthma. We constructed a mouse model of ovalbumin-induced AA and overexpressed IFN-*γ* to evaluate the effect on the IL-27/Th9 axis via the in vitro effect of IFN-*γ* on IL-27 secretion by DCs and their influence on Th9 differentiation and asthmatic inflammation. IFN-*γ* overexpression reduced the proportion of Th9 cells and DCs and altered lung morphology and cytokine production in AA-induced mice, thus suppressing the AA phenotype. In addition, exogenous IFN-*γ* stimulation promoted the secretion of IL-27 and suppressed Th9 differentiation of CD4+ T cells via signal transducer and activator of transcription 1/3 (STAT1/3) signaling in a time-dependent manner. This study aimed to clarify the regulatory effect and mechanism of the IFN-*γ*/DCs/IL-27/Th9 axis on AA and provide novel insights for effective targeted treatment of asthma.

## 1. Introduction

Allergic asthma (AA) is a chronic inflammatory airway disease triggered by immunogen sensitization and is manifested by symptoms such as shortness of breath, coughing, and chest tightness. AA is one of the most common respiratory diseases affecting over 300 million people worldwide and has become a challenging public health problem that severely diminishes quality of life and causes socioeconomic loss [1]. Clinically, anti-AA agents such as systemic steroid hormones, bronchodilators, *β*-receptor blockers, leukotriene receptor blockers, and antihistamines form the cornerstones of AA treatment and are currently widely adopted [2–4]. Although these methods are highly successful in managing symptoms of AA, adverse side effects are common and inflammation is not completely controlled [5–7]. Consequently, there is an increasing demand to improve current techniques or develop new ways of effectively treating asthma. In doing so, significant focus must be placed on understanding the molecular pathogenesis of AA.

Several cytokines have been highlighted as targets in asthma research because of their putative roles in regulating the immune response and inflammation [8]. Interleukin (IL)-9 is a pleiotropic cytokine that is abundantly expressed in Th2 inflammation-based diseases. Although IL-9 was originally thought to be a Th2 cytokine [9], later studies suggested that it is mainly secreted by Th9 cells, which are considered as a new T cell subgroup [10, 11]. Th9 cells play a critical role in the initiation and progression of inflammation in asthma. IL-27 is a member of the IL-12 family and is a heterodimer with IL-27R (composed of IL-27R*α* and the gp130 protein complex) as its receptor [12]. IL-27 is mainly expressed in activated macrophages and dendritic cells (DCs), whereas IL-27R is widely expressed in T cells, natural killer cells, monocytes, mast cells, endothelial cells, activated B cells, and DCs [13]. IL-27 elicits different responses from a range of T cell subtypes and can promote a Th1 response while suppressing a Th2 response and production of Th2 cytokines, thereby inhibiting the Th17 response [13, 14]. Importantly, IL-27 can inhibit Th9-driven differentiation of CD4+ T cells, a process that depends on signal transducer and activator of transcription (STAT) and T-bet signaling [15]. The therapeutic application of IL-27 has been explored in treating a variety of diseases, such as allergic inflammation, arthritis, and encephalomyelitis. Although the Th9 axis plays an important part in the appearance and persistence of asthma, the regulatory mechanisms remain poorly understood. Similarly, the expression, distribution, and upstream regulation of IL-27 in asthma and regulation of the Th9 response, which plays a vital role in the pathogenesis of asthma, remain unreported.

The role of interferon (IFN)-*γ* in asthma has been debated because, like IL-9, this has pleiotropic roles in influencing the properties and functions of target cells. Although the proinflammatory effects of IFN-*γ* have been widely demonstrated, this has also been shown to inhibit Th2 cell proliferation [16]. In rhinovirus-infected mice, the type 2 immune response representing an asthmatic phenotype was suppressed by IFN-*γ*, which was shown by the inhibition of type 2 innate lymphoid cell expansion and attenuation of mucous metaplasia [17]. A variety of factors contribute to the differential function of IFN-*γ*, such as dose and cell-specific interactions [18]. The regulatory effect of IFN-*γ* on asthmatic inflammation and its relationship with IL-27 and Th9 response have prominent practical significance for AA treatment and need to be elucidated.

Herein, we speculated that IFN-*γ* can inhibit Th9 differentiation by regulating the secretion of IL-27 by DCs, thereby suppressing airway inflammation in asthma. We constructed a mouse model of ovalbumin-induced AA and overexpressed IFN-*γ* to evaluate the effect on the IL-27/Th9 axis. We investigated the in vitro effect of IFN-*γ* on IL-27 secretion by DCs and their influence on Th9 differentiation and asthmatic inflammation. The objective of this study was to clarify the impact and mechanism of regulation of the IFN-*γ*/DC/IL-27/Th9 axis on AA, providing novel insights for the effective targeted treatment of asthma.

## 2. Materials and Methods

### 2.1. Ovalbumin-Induced Animal Model of AA

In vivo experiments were performed at the Model Animal Research Institute at Wuhan Myhalic Biotechnology Co., Ltd. (Wuhan, China). The study was approved by the institutional review board and adhered to the “Guidelines for Animal Care and Use of the Model Animal Research Institute at Wuhan Myhalic Biotechnology Co., Ltd.” (approval number HLK-20190310-01). The animal model of AA was constructed via ovalbumin induction. Twenty-four female specific-pathogen-free C57BL/6 mice (weighing 19–21 g, aged 2–3 months) were randomly divided into four groups (*n* = 6 per group): control (no treatment); AA (ovalbumin induction); AA + NC (ovalbumin induction with negative control transfection); and AA + OV-IFN-*γ* (ovalbumin induction with IFN-*γ* overexpression). Prior to OVA induction, 40 *μ*g of ovalbumin (SLBQ9036V, Sigma-Aldrich, St. Louis, MO) and 2 mg of aluminum hydroxide (239186, Sigma-Aldrich) were mixed in 200 *μ*L of sterilized phosphate-buffered saline (PBS). The ovalbumin mixture was injected intraperitoneally on days 1 and 14. Mice in the AA + NC and AA + OV-IFN-*γ* groups were transfected with 10 *μ*g of NC or OV-IFN-*γ* vectors, respectively, via tail vein injection on day 26 and every three days thereafter (on day 29 and day 32). From day 28 to day 31, nebulization was performed daily with 5% OVA for 30 min, after which 20 *μ*L of ovalbumin was injected into the nose of the animals at 40 mg/mL. On day 32, mice were sacrificed by cervical dislocation. Animal Model of AA and treatment in graphic abstract (Figure 1).

### 2.2. IFN-*γ* Overexpression Vector Construction

To overexpress IFN-*γ*, the overexpression fragment (forward: GCTCTAGATGAACGCTACACACTGC;

reverse: CGGGATCTCAGCAGCGACTCCTTTT) was inserted into the pCDH-CMV-MCS-EF1-CopGFP-T2A-Puro vector (Addgene, Watertown, MA), with XhoI and BamHI restriction sites. Vectors were transfected into HEK293T cells (GNHu17, provided by the cell bank of the Chinese Academy of Sciences) for 24 h [19], after which the transfection efficiency was determined by quantitative reverse transcription polymerase chain reaction (qRT-PCR) and western blot.

### 2.3. Sample Collection

Serum bronchoalveolar lavage fluid (BALF) and lung tissue were collected. Whole blood was extracted from the eyes of the mice before sacrifice. Briefly, mice were anesthetized with an intraperitoneal injection of 1% sodium pentobarbital at 40 mg/kg. After full anesthesia, 1 mL of orbital blood was collected by inserting capillaries into blood vessels beneath the eye. Half of the blood sample was stored for flow cytometry analysis, and the other half was separated by centrifugation at 5000 rpm for 20 min to obtain serum for cytokine production analysis. To extract BALF, precooled sterile PBS was injected via tracheal intubation. The tube was withdrawn three times, and BALF was obtained each time, with a recovery rate of above 90%. Half of the BALF sample was filtered with a steel mesh, washed twice, and resuspended in RPMI 1640 medium at a density of 5 × 10^6^ cells/mL. Monocytes and macrophages were removed by the adherence method, and the remaining cells were stored for flow cytometry analysis. The other half of the BALF sample was centrifuged at 1500 rpm for 10 min, after which the supernatant was stored at −80 °C for cytokine detection. After blood collection and BALF extraction, the mice were sacrificed by cervical dislocation. To extract lung tissue, the mice were dissected following sacrifice, and 5 mL of saline was injected into the right ventricle to flush out the blood in the lung. Tissues from the lavage right lung were homogenized, and the supernatant was collected for cytokine detection. The left lung was fixed with 4% paraformaldehyde and used for histological analysis.

### 2.4. Isolation and Culture of Bone Marrow-Derived DCs [20, 21]

Healthy male C57BL/6 mice (aged 8–12 weeks) were sacrificed by cervical dislocation and immersed in 75% ethanol for 5 min. The femur and tibia were extracted in an aseptic environment and immersed in RPMI 1640 medium. Culture medium was aspirated using a syringe, and the bone marrow cavity was pierced from one end. The medium was injected so that the marrow was flushed into a Petri dish. The marrow was washed repeatedly, and the resulting cell suspension was centrifuged for 10 min at 1500 rpm. Supernatant was removed, and 3 mL of sterile red blood cell lysis solution (NH4CL2009, TBD Science, Tianjin, China) was added to lyse the bone marrow-derived red blood cells at room temperature for 2 min. Then, 5 mL of RPMI 1640 medium was added, and the cell suspension was centrifuged for 5 min at 1500 rpm. Supernatant was removed, and the cells were washed once with RPMI 1640 medium and centrifuged again for 5 min at 1500 rpm. Supernatant was removed, and cells resuspended and seeded in a 6-well plate with 4 mL of medium in each well containing 20 ng/mL recombinant mouse granulocyte-macrophage colony-stimulating factor (415-ML-005, R&D Systems) and 10 ng/mL IL-4 (51084-MNAE, Sino Biologicals Inc., North Wales, PA). Cells were cultured in the absence of serum for 48 h at 37 °C and 5% CO_2_. To obtain DC-conditioned medium, cells were centrifuged at 400×*g* for 15 min to separate cells and cell fragments from the medium, and the extracted medium was filtered using a 0.22-*μ*m filter.

### 2.5. Isolation and Th9 Induction of Spleen-Derived CD4+ T Cells [22]

CD4+ T cells were isolated from the spleen using a specialized reagent kit (LTS1092PK, TBD Science). Spleen tissues were ground and passed through a 200-mesh filter, and the supernatant was collected from the ground tissues. After centrifugation, 2 mL of erythrocyte lysate was added into the supernatant. When the lysis solution was cleared, a two-fold volume of PBS was added to end lysis. The suspension was centrifuged, and the precipitated cells were washed with PBS. Cells were resuspended in flow cytometry buffer at 2 × 10^7^cells/mL, and an equal volume of separation fluid was added. The single-cell suspension was carefully aspirated to the top of the liquid and centrifuged for 30 min at 400×*g*. After centrifugation, the liquid in the tube was separated into four layers. The milky ring-shaped layer of lymphocytes (second layer) was aspirated to a new tube with 10 mL of wash buffer (2010X1118, TBD Science). After 10 min of centrifugation at 250×*g*, remove the supernatant, and add 5 mL of wash buffer with the cells centrifuged again for 10 min at 250×*g*. Isolated cells were identified as CD4+ T cells using flow cytometry. To induce Th9 differentiation, isolated CD4+ T cells were seeded in a culture plate precoated with 2 *μ*g/mL CD3 antibody (ab16669, Abcam) and 2 *μ*g/mL CD28 antibody (ab213043 Abcam), with 50 *μ*M 2-mercaptoethanol, RPMI 1640 medium containing 5% fetal bovine serum, 1% penicillin/streptomycin and 1% L-glutamine, pyruvate, and 50 *μ*M 2-mercaptoethanol. Three days after differentiation, cells were stimulated with 20 ng/mL il-4 (51084-mnae, Sino biological Inc.) and 3ng /mL transforming growth factor (TGF)-*β* (50698-m08h, Sino biological Inc.) for 48 h. Cells were collected and CD4 + IL-9+ (Th9) cells were identified by flow cytometry.

### 2.6. Quantitative Real-Time PCR (qRT-PCR) [23]

Tissue or cell samples were homogenized with 1 mL of TRIzol reagent for RNA extraction. Reverse transcription using the Advantage® RT-for-PCR Kit (Takara, Kyoto, Japan), and qRT-PCR was performed using the SYBR Green PCR kit (KAPA Biosystems, Wilmington, MA) on a CFX-Connect 96 system (Bio-Rad, Hercules, CA). The mRNA primers are shown in Table 1. The data were analyzed using the 2^-*ΔΔ*Ct^ method. Reaction conditions were as follows: initial denaturation at 95 °C for 3 min; 39 cycles of denaturation at 95 °C for 5 s, annealing at 56 °C for 10 s, and extension at 72 °C for 25 s; and final extension at 65 °C for 5 s and 95 °C for 50 s.

### 2.7. Western Blot [24]

Samples were cleaved to collect proteins. For western blot, proteins were first denatured by boiling for 10 min. Then, 20 *μ*g of protein sample was loaded onto a 12% polyacrylamide gel for sodium dodecyl sulfate-polyacrylamide gel electrophoresis at 120 V for 50 min. Separated proteins were transferred onto polyvinylidene fluoride membranes (presoaked in acetone for 5 min) at 90 V for 50 min. Membranes were blocked with 5% skim milk overnight at 4 °C and incubated overnight at 4 °C with antibodies against the proteins of interest listed in Table 2. After three washes with PBS/Tween for 5 min each, the membranes were incubated at room temperature for 1 h with secondary antibodies and washed again three times. Membranes were then immersed in an enhanced chemiluminescence reaction solution in the dark, and the protein bands were scanned using a Tanon-5200 automatic analyzer (Tanon, Shanghai, China). Band gray values were analyzed using Tanon GIS software [19].

### 2.8. DCs Were Detected by Flow Cytometry

Cells were resuspended in flow cytometry buffer with phycoerythrin-conjugated antibodies to CD11c (85-12-0114-81, eBioscience, San Diego, CA, USA) and incubated for 30 min at 4 °C in the dark. Flow cytometry buffer was added, and cells were centrifuged for 5 min at 4 °C at 300×*g*. The supernatant was removed, and the cells were resuspended in flow cytometry buffer. Flow cytometry was performed using a NovoCyte apparatus (ACEA Biosciences, San Diego, CA), and the data were analyzed using built-in software.

### 2.9. CD4+/IL-9+ (Th9) T Cells Were Detected by Flow Cytometry [23]

Cells were resuspended in culture medium containing 50 ng/mL Leukocyte Activation Cocktail (550583, BD Bioscience, Franklin Lakes, NJ, USA), 2 *μ*g/mL ionomycin (I8800, Solarbio, Beijing, China), and 3 *μ*g/mL monensin sodium (M8670, Solarbio) and incubated for 6 h at 37 °C in an atmosphere containing 5% CO_2_. Cells were then washed with flow cytometry buffer and centrifuged for 5 min at 4 °C at 300×*g*. Supernatant was discarded, and cells were incubated in flow cytometry buffer containing fluorescein isothiocyanate-conjugated antibodies to CD4 (85-11-0041-81, eBioscience) for 30 min at 4 °C. Cells were then incubated with permeabilization buffer for 20 min and centrifuged for 5 min at 4 °C at 300×*g*, after which the supernatant was discarded. Flow cytometry buffer containing eFluor 660-conjugated antibodies against IL-9 (85-50-8091-80, eBioscience) was added to the cells and incubated for 45 min at 4 °C. Cells were resuspended in flow cytometry buffer, and flow cytometry and data analysis were performed using NovoCyte apparatus and software.

### 2.10. Histological Analysis

Lung tissues were cut into small pieces, dehydrated, and embedded in paraffin wax. The tissue block was cooled at −20 °C and sectioned at 4 *μ*m; tissue sections were transferred to a glass slide for staining.

### 2.11. Hematoxylin/Eosin Staining [23]

Tissue sections were dehydrated and washed with water. After 5 min of staining in hematoxylin solution (I1709, Bioswamp, Wuhan, China), the residual dye was removed by washing the sections with running water for 2 min. Sections were then immersed in 1% hydrochloric acid alcohol for 3 s, washed with water for 2 s, and immersed in bluing solution for 10 s. Sections were stained with 0.5% eosin solution (I1703, Bioswamp), washed with distilled water, and immersed in increasing concentrations of ethanol. After one dip in anhydrous ethanol and two washes with xylene, the sections were sealed with neutral balsam gum and observed using an optical microscope.

### 2.12. Masson's Trichrome Staining

Masson's trichome staining was performed using an assay kit (K1812, Bioswamp), and all reagents were included in the kit. Tissue sections were dehydrated and stained for 10 min with a solution composed of equal volumes of hematoxylin and ferric chloride solution. Sections were then differentiated using an ethanol hydrochloride differentiation solution and blued using an ammonia solution. After 1 min of washing with deionized water, the sections were dyed in a Ponceau acid fuchsin solution for 5 min and immersed in an aqueous solution of acetic acid for 1 min, an aqueous solution of phosphomolybdic acid for 2 min, and an aqueous solution of acetic acid for 1 min. Thereafter, sections were stained in an aniline blue solution for 2 min and immersed in an aqueous solution of acetic acid for 1 min. Sections were quickly dehydrated using ethanol and in xylene. Sealed and observed.

### 2.13. Alcian Blue/Periodic Acid-Schiff (AB/PAS) Staining

AB/PAS staining was performed using an assay kit (K1932, Bioswamp), and all reagents were included in the kit. Tissue sections were dehydrated and stained for 5 min with Alcian blue solution. After 2 min of washing with tap water, sections were stained for 15 min with periodic acid solution and washed once with tap water and twice with distilled water. Then, the sections were stained for 30 min with Schiff dye solution in the dark. After hematoxylin, washed with anhydrous ethanol, and transparentized with xylene. Seal with neutral resin and observe with inverted microscope.

### 2.14. Semi-Quantitative Analysis of Histological Staining

Semi-quantitative analysis staining was using Image-Pro Plus 6.0 (Media Cy). Areas of inflammatory infiltration were identified as positive staining. Blue area indicative of collagen deposition was identified as positive staining. Light magenta area indicative of mucin production was identified as positive staining. The positive area for each staining was normalized to and expressed as a percentage of the total staining area.

### 2.15. Enzyme-Linked Immunosorbent Assay (ELISA)

Secretion of the following cytokines was evaluated using the corresponding ELISA kits from Bioswamp (Wuhan, China): IFN-*γ* (MU30038-S), IL-27 (MU30243), IL-27R (MU30868), IL-9 (MU30658), and IL-6 (MU30044). Culture medium was collected and added to the wells of a 96-well plate that had been precoated with antibodies against the cytokine of interest. Biotinylated antibodies were added, followed by the addition of horseradish peroxidase-conjugated solution. The plate was then incubated at 37 °C for 30 min, and chromogen was added for 10 min. Add stop solution to stop the reaction, and the absorbance of the wells was measured at 450 nm using a microplate reader.

### 2.16. Statistical Analysis

All tests were done in three technical replicates from pooled samples of three cell samples (*n* = 3) or six animals (*n* = 6) per group for in vitro and in vivo studies, respectively. All statistical analysis was performed using OriginPro 8.0 (OriginLab). The data are presented as *mean* ± *standard* *deviation*. One-way analysis of variance followed by Tukey's post hoc test was performed to evaluate the significance of the difference between mean values. A *p* value of <0.05 indicated statistical significance.

## 3. Results

### 3.1. The Transfection Efficiency of the IFN-*γ* Overexpression (OV-IFN-*γ*) Vector

We first investigated whether IFN-*γ* overexpression influenced the production of Th9 cells and DCs in AA-induced mice. The transfection efficiency of the IFN-*γ* overexpression (OV-IFN-*γ*) vector was first confirmed in HEK293T cells by qRT-PCR (Figure 2(a)) and western blot (Figure 2(b)), which showed that transfection IFN-*γ* overexpression plasmid induced significantly greater expression of *IFN-γ* mRNA compared with that in non-transfected cells and those transfected with negative control (NC) vectors (empty vectors).

### 3.2. IFN-*γ* Overexpression Reduced the Proportion of Th9 Cells and DCs in Ovalbumin-Induced Mice

Ovalbumin-induced mice (AA model) were then transfected with NC or OV-IFN-*γ* vectors, and flow cytometry was carried out to examine the proportion of Th9 cells (CD4+ T cells positive for IL-9) (Figure 3) and DCs (positive expression of CD11c) (Figure 4) in peripheral blood and BALF. In both peripheral blood and BALF, AA-induced mice contained a significantly greater percentage of cells expressing IL-9 or CD11c compared with that in control mice. The NC had no effect on AA-induced mice, whereas OV-IFN-*γ* transfection led to significant decreases in the percentages of IL-9+ and CD11c + cells in peripheral blood and BALF. This indicates that AA triggered an increase in the production of Th9 cells and DCs, but populations of these cells were reduced by OV-IFN-*γ*.

### 3.3. IFN-*γ* Altered Lung Morphology in Ovalbumin-Induced Mice

We then evaluated whether IFN-*γ* overexpression affected lung morphology and cytokine production in AA-induced mice. First, H&E staining (Figure 5(a)) revealed that the subepithelial layers of the lung tissues were thickened in AA-induced mice, with clear signs of inflammatory infiltration (black arrows). Masson's trichrome staining (Figure 5(b)) revealed a substantial amount of collagen deposition (black arrows pointing to blue areas), while AB/PAS staining (Figure 5(c)) indicated the presence of excess mucin production (black arrows pointing to light magenta areas) in the lungs of AA-induced mice. In all cases, the NC did not exert an apparent effect on lung morphology. However, based on histopathological observations, AA-induced mice that were transfected with OV-IFN-*γ* vectors showed improvements in lung morphology. In particular, inflammatory infiltration was alleviated, collagen deposition was suppressed, and mucin production was reduced.

### 3.4. IFN-*γ* Altered Cytokine Production in Ovalbumin-Induced Mice

Next, as we were interested in the effect of IFN-*γ* on IL-27 activity, we assessed the expression of mRNA of *IL-27* and the associated receptor *IL-27R* in the lungs of AA-induced mice (Figure 6(a)). Compared with that of the control mice, ovalbumin induction caused a significant decrease in the expression of both *IL-27* and *IL-27R* mRNA, which was recovered by OV-IFN-*γ* transfection. We then examined the secretion of various cytokines in the lung, serum, and BALF samples (Figure 6(b)). Ovalbumin induction led to a significant decrease in the expression of IFN-*γ*, IL-27, and IL-27R and a significant increase in the expression of IL-9 and IL-6 in the lung, serum, and BALF of mice. However, transfection with OV-IFN-*γ* reversed the effect of ovalbumin by upregulating IFN-*γ*, IL-27, and IL-27R expression and downregulating IL-9 and IL-6 expression. In all cases, the NC vectors did not exert any significant difference in cytokine expression.

### 3.5. Effect of Exogenous IFN-*γ* Stimulation on IL-27 Expression in DCs and Th9 Cell Phenotype

Next, we investigated whether exogenous IFN-*γ* stimulation could affect the properties of DCs and CD4+ T cells isolated from mice. DCs were extracted from the bone marrow of C57BL/6 mice, and their purity was verified by assessing the percentage of CD11c + cells [25] by flow cytometry (Figure 7(a)). Isolated DCs were stimulated by recombinant mouse IFN-*γ* at 100 ng/mL, and the expression of *IL-27* mRNA and the expression of secretion of IL-27 protein were evaluated (Figures 7(b)–7(d)). Compared with unstimulated DCs, cells stimulated with recombinant IFN-*γ* exhibited significantly higher expression of IL-27 both transcriptionally and as a secreted protein.

Subsequently, we isolated CD4 + CD62L + CD44- T cells from the spleen of C57BL/6 mice and induced their differentiation into the Th9 phenotype in vitro. Th9 cells were stimulated with recombinant mouse IFN-*γ* at 100 ng/mL, and changes in the Th9 phenotype were observed. Flow cytometry sorting revealed that Th9-specific medium induced a large increase in the proportion of IL-9-positive (Th9-differentiated) CD4+ T cells, indicating the successful induction of Th9 differentiation (Figure 8(a)). qRT-PCR and ELISA, respectively, demonstrated that the expression of *IL-9* mRNA and secretion of IL-9 protein in IFN-*γ*-stimulated Th9 cells was significantly suppressed compared with that in unstimulated cells (Figures 8(b) and 8(c)). IFN-*γ* stimulation at 100 ng/mL also significantly elevated the expression of *T-bet* mRNA, a Th1-specific transcription factor [26], in a time-dependent manner for up to 120 min (Figure 8(d)), suggesting a shift in CD4+ T cells toward the Th1 phenotype.

In terms of molecular mechanism, we examined whether exogenous IFN-*γ* stimulation affected the STAT1/STAT3 signaling pathway in Th9 cells (Figure 8(e)). The phosphorylation level of STAT1 relative to total STAT1 protein expression was increased by IFN-*γ* stimulation in a time-dependent manner. However, STAT3 phosphorylation (relative to total STAT3 protein expression) showed a time-dependent decrease upon IFN-*γ* stimulation. The results reflect the state of Th9 cells for up to 120 min, and there appeared to be no significant difference between 20 and 60 min of stimulation.

### 3.6. DC-Conditioned Medium Affected Cytokine Production and T Cell Phenotype

Based on the premise that IFN-*γ* stimulation induced the secretion of IL-27 from DCs, we investigated whether DC culture media contains factors that affect Th9 cells. Spleen-derived CD4+ T cells were Th9-differentiated and cultured for 72 h with conditioned medium collected from either unstimulated or IFN-*γ*-stimulated DCs. Thereafter, the secretion of IFN-*γ*, IL-27, and IL-9 from Th9 cells was measured. Compared with Th9 cells cultured in normal medium, those cultured with conditioned medium from unstimulated DCs showed elevated secretion of IFN-*γ* and IL-27, but without any change in IL-9 secretion (Figure 9(a)). However, when Th9 cells were cultured with medium from IFN-*γ*-treated DCs, IFN-*γ* and IL-27 secretion were further promoted, whereas IL-9 secretion was suppressed. We also measured the expression of *IL-9* and *T-bet* mRNA after culturing Th9 cells with DC-conditioned medium (Figure 9(b)). Consistent with these results, the expression of *IL-9* mRNA was unchanged by conditioned medium from unstimulated DCs but was significantly reduced by conditioned medium from IFN-*γ*-stimulated DCs. However, whereas the expression of the Th1-specific *T-bet* mRNA was unaffected by conditioned medium from unstimulated DCs, this was significantly increased by the addition of conditioned medium from IFN-*γ*-stimulated DCs to Th9 cells.

### 3.7. DC-Conditioned Medium Exhibited Time-Dependent Effects on STAT1/STAT3 Signaling in Th9 Cells

We performed western blot analysis to verify whether the effect of IFN-*γ* stimulation in DCs on the STAT signaling pathway could be transferred to Th9 cells during co-culture with conditioned medium (Figure 10(a)). In Th9 cells cultured under normal conditions (no addition of DC-conditioned medium), the phosphorylation levels of STAT1 (Figure 10(b)) and STAT3 (Figure 10(c)), relative to the total expression of the respective protein, were unchanged for up to 120 min. The same was observed for Th9 cells cultured with conditioned medium from unstimulated DCs, where minimal changes were detected over time. However, conditioned medium from IFN-*γ*-stimulated DCs caused a time-dependent increase in phosphorylation of STAT1 and a time-dependent decrease in STAT3 phosphorylation. In addition, at each time point of culture duration (20, 60, and 120 min), the expression of p-STAT1/STAT1 was higher and that of p-STAT3/STAT3 was lower in Th9 cells cultured in conditioned medium from IFN-*γ*-stimulated DCs compared with the expression in cell culture under normal conditions.

## 4. Discussion

The pathogenesis of AA is thought to implicate a type 2 immune response, involving the production of cytokines such as IL-4, IL-5, and IL-13 [27]. This results in an asthmatic phenotype of airway inflammation, mainly in the form of airway hyperresponsiveness and tissue remodeling [28]. Initiation and progression of AA are associated with a complex interconnection between inflammation and immune response [29, 30]. Altered inflammatory signaling cascades may induce changes in the immune response and vice versa. Thus, a thorough understanding of the interaction between inflammatory and immunomodulatory factors involved in the pathogenesis of AA is crucial for the development of anti-asthma targeted therapies. This study reports specific interactions underlying the molecular action of IFN-*γ* in AA regulation as outlined in Figure 11.

The participation of IFN-*γ* in mediating inflammation has gained attention in recent asthma-related research. In autoimmune encephalomyelitis, IFN-*γ* reportedly inhibits Th9-mediated autoimmune inflammation by regulating DC secretion of IL-27. In vivo and in vitro studies have also demonstrated that IFN-*γ* induces the production of IL-27 by DCs and inhibits osteopontin expression, thereby suppressing IL-17-mediated autoimmune inflammation. In addition, the combination of IFN-*γ* and IL-27 can alter the function of type 2 innate lymphoid cells via STAT1-dependent mechanisms. In a mouse model of asthma, administration of IFN-*γ* into the nasal cavity suppressed the allergic inflammatory response in the lungs, ameliorated the symptoms of AA, and reduced eosinophil accumulation [31]. Our results on IFN-*γ* in an AA mouse model are consistent with those of previous studies, wherein IFN-*γ* overexpression alleviated the asthmatic pulmonary phenotype by attenuating inflammatory infiltration, collagen fiber deposition, and mucus production in the lungs of AA-induced animal. In addition, IFN-*γ* overexpression promoted the secretion of IL-27 and IL-27R while inhibiting that of IL-9 in the lung, serum, and BALF of AA-induced mice, consistent with previous studies.

We note more interestingly that the increase in DC proportion induced by the AA phenotype was suppressed by IFN-*γ* overexpression, with further implications on the immune response. DCs are the main antigen-presenting cells in the immune system and play an important role in mediating pulmonary inflammation during AA [32, 33]. DCs are critically involved in the differentiation of CD4+ T cells by producing cytokines such as IL-27 [34]. Research on the role of IL-27 in asthma has indicated that IL-27 may increase the expression of *T-bet* mRNA by promoting IFN-*γ* expression, inhibiting IL-4 synthesis, and enhancing the Th1 response [35, 36]. The way IL-27 regulates T cell immunity is complex. IL-27 can act as a proinflammatory factor, but this also exhibits anti-inflammatory effects [37, 38]. IL-27 was demonstrated to inhibit the differentiation of FOXP3+ Treg cells through a STAT3-dependent mechanism [39]. Other studies have also revealed that IL-27 mediates the production of IL-10 by T cells through STAT-related signaling [40, 41]. Activation of STAT signaling by IL-27-mediated regulation was further demonstrated in CD8+ T cells [42, 43].

Th9 immune response has been implicated in a variety of inflammation-related diseases and autoimmune diseases [44]. In asthma, IL-9 appears to promote the proliferation of activated T cells and production of IgE by B cells [45]. Production of IL-9 by activated CD4+ T cells can be enhanced by TGF-*β* and IL-4 but is blocked by IFN-*γ* [46]. Upon antigen stimulation, IL-9 secreted by Th9 cells also regulates the number of mast cells and triggers tissue remodeling during inflammation [47]. A recent study with adoptive transfer of Th9 or Th2 cells to Rag2^−/−^ mice showed that the Th9 response is more effective than that of Th2 in causing severe asthma symptoms [48]. The link between Th9 differentiation and STAT signaling has also been demonstrated. Th9 differentiation was associated with normal phosphorylation of STAT3, which in turn correlates with impaired STAT1 phosphorylation/activation and suppressed transcription of *T-bet* [49].

Based on the collective evidence of the correlation between Th9, IL-27, and STAT signaling, we evaluated whether IFN-*γ*-induced IL-27 production in DCs is associated with STAT activation and Th9 differentiation. Our results revealed the following: (1) In the AA model, IFN-*γ* inhibited Th9 cell and DC recruitment while alleviating the symptoms and phenotype of AA; (2) in vitro, IFN-*γ* stimulation promoted the production of IL-27 from DCs and inhibited the release of IL-9 from CD4+ T cells via STAT1/3-mediated signaling; and (3) when cultured with conditioned medium from IFN-*γ*-stimulated DCs, CD4+ T cells showed a decrease in the Th9 phenotype, which was mediated by STAT1/3 signaling. These results suggest that IFN-*γ* indirectly acts on CD4+ T cells by triggering IL-27 production by DCs, and IL-27 in conditioned medium in turn stimulates CD4+ T cells to alter their phenotype. This is manifested as an increase in Th1-specific response (increased *T-bet* mRNA expression) and a decrease in Th9-specific response (decreased expression of *IL-9* mRNA and decreased secretion of IL-9 protein). There was also a clear time-dependent effect on STAT1/3 signaling. This is consistent with previous studies reporting that IFN-*γ* is associated with induction (phosphorylation) of STAT1 [50] and dephosphorylation of STAT3 [51]. The opposing effects of STAT1 and STAT3 have also been demonstrated in previous reports [52, 53], further supporting the results of our study. We note here that STAT1/3 is by no means the only signaling pathway that exerts an effect on IFN-*γ*-mediated immune response, but one of many that may partly contribute to the function of IFN-*γ*. Other important signaling pathways, such as phosphatidylinositol-4,5-bisphosphate 3-kinase/mammalian target of rapamycin [54] and nuclear factor-kappaB [55], may influence the effect of IFN-*γ*. Here, we chose to focus on STAT signaling because although an involvement in the Th9 response has been suggested, further molecular implications are lacking. Our findings provide insight into the relationship between Th9 and STAT signaling, but further studies are required to elucidate the role of other signaling pathways in Th9-mediated AA.

Our study has several limitations that will be addressed in future studies. First, we did not carry out an in-depth comparison between the roles of Th2 and Th9. Although a previous study showed that the Th9 response was stronger than the Th2 response in asthma [23], without further research, we cannot definitively say whether the Th9 or Th2 response is stronger upon IFN-*γ* stimulation because of the complex interplay between immune factors and the pleiotropic functions of IFN-*γ* and Th9 cells. In addition, whereas the time-dependent effect of IFN-*γ* was studied here, the concentration-dependent effects may also be of particular interest. The concentration of IFN-*γ* has been heavily implicated in associated functions in previous reports, and therefore, a more comprehensive understanding of the regulatory role of IFN-*γ* will require studies that test a minimum of three concentrations. Furthermore, in this study, the use of DC-conditioned medium was sufficient to elucidate the effect of DC-secreted factors on Th9 differentiation of CD4+ T cells. However, direct co-culture of DCs and CD4+ T cells, ideally in a three-dimensional microenvironment that mimics the inflammatory/immune niche, will represent an authentic scenario in vivo more accurately. Prospective research will consider these factors to improve the study design.

Based on the results of this study, we clarified the molecular mechanisms implicated in the involvement of IFN-*γ* in AA regulation. We propose that IFN-*γ* stimulates the release of IL-27 from DCs, which in turn inhibits the Th9 differentiation of CD4+ T cells to alleviate the AA phenotype. These findings provide critical insights into the collaborative actions of various components of the immune/inflammatory axis and contribute to the future research and development of therapeutic schemes to treat AA.

## Figures and Tables

**Figure 1:** Graphic abstract.

**Figure 2:** The transfection efficiency of the IFN-*γ* overexpression (OV-IFN-*γ*) vectors. (a) qRT-PCR and (b) western blot analysis of transfection efficiency of IFN-*γ* overexpression vectors evaluated in HEK293T cells. Control represents non-transfected cells and negative control represents transfection of empty vectors. Results are presented as *mean* ± *SD* (*n* = 3), ∗*p* < 0.05.

**Figure 3:** Flow cytometry analysis and quantification of the proportion of Th9+ cells in peripheral blood and BALF of ovalbumin-induced (AA) mice, with or without NC/OV-IFN-*γ* transfection. Results are presented as *mean* ± *SD* (*n* = 6), ∗*p* < 0.05. Control represents non-AA mice. IFN: interferon; AA: allergic asthma; NC: negative control; ov: overexpression; BALF: bronchoalveolar lavage fluid.

**Figure 4:** Flow cytometry analysis and quantification of the proportion of CD11c + (dendritic) cells in peripheral blood and BALF of ovalbumin-induced (AA) mice, with or without NC/OV-IFN-*γ* transfection. Results are presented as *mean* ± *SD* (*n* = 6), ∗*p* < 0.05. Control represents non-AA mice. IFN: interferon; AA: allergic asthma; NC: negative control; ov: overexpression; BALF: bronchoalveolar lavage fluid.

**Figure 5:** IFN-*γ* altered lung morphology in ovalbumin-induced mice. (a) H&E, (b) Masson's trichrome, and (c) AB/PAS staining of lung tissues in ovalbumin-induced (AA) mice, with or without NC/OV-IFN-*γ* transfection. Corresponding quantification of staining is shown in bar charts in terms of area %. Black arrows point to areas of inflammatory infiltration in H&E staining, collagen deposition (blue) in Masson's trichrome staining, and mucin production (light magenta) in AB/PAS staining. *Scale* *bar* = 50 *μm*.

**Figure 6:** IFN-*γ* altered cytokine production in ovalbumin-induced mice. (a) qRT-PCR analysis of expression of *IL-27* and *IL-27R* mRNA in lung tissues of ovalbumin-induced (AA) mice, with or without NC/OV-IFN-*γ* transfection. (b) ELISA of secreted IFN-*γ*, IL-27, IL-27R, IL-9, and IL-6 in lung homogenate, serum, and BALF of ovalbumin-induced (AA) mice, with or without NC/OV-IFN-*γ* transfection. Results are presented as *mean* ± *SD* (*n* = 6), ∗*p* < 0.05. Control represents non-AA mice. IFN: interferon; AA: allergic asthma; NC: negative control; ov: overexpression; IL: interleukin; H&E: hematoxylin and eosin; AB/PAS: Alcian blue/periodic acid-Schiff; BALF: bronchoalveolar lavage fluid.

**Figure 7:** Characterization of isolated DCs stimulated with IFN-*γ*. DCs were extracted from bone marrow of C57BL/6 mice and stimulated with 100 ng/mL IFN-*γ*. (a) Flow cytometry validation of successful isolation of DCs. Cells expressing CD11c were identified as DCs. (b) qRT-PCR analysis of expression of *IL-27* mRNA in unstimulated and IFN-*γ*-stimulated DCs. (c) ELISA of secreted IL-27 in unstimulated and IFN-*γ*-stimulated DCs. (d) Western blot analysis and quantification of IL27 protein expression in unstimulated and IFN-*γ*-stimulated DCs. Results are presented as *mean* ± *SD* (*n* = 3), ∗*p* < 0.05. DCs: dendritic cells; IL: interleukin.

**Figure 8:** Characterization of isolated CD4+ T cells stimulated with IFN-*γ*. CD4+ T cells were extracted from the spleen of C57BL/6 mice and stimulated with 100 ng/mL IFN-*γ* for 20, 60, or 120 min. (a) Flow cytometry validation of T cell differentiation into Th9 subset with or without IFN-*γ* stimulation. Cells expressing IL-9 were identified as Th9 cells. (b) qRT-PCR analysis of expression of *IL-9* mRNA in unstimulated and IFN-*γ*-stimulated T cells. (c) ELISA of secreted IL-9 in unstimulated and IFN-*γ*-stimulated T cells. (d) qRT-PCR of expression of *T-bet* mRNA in unstimulated and IFN-*γ*-stimulated (20, 60, or 120 min) T cells. (e) Western blot analysis and quantification of the phosphorylation of STAT1 and STAT3 (relative to total protein content) in unstimulated and IFN-*γ*-stimulated (20, 60, or 120 min) T cells. Results are presented as *mean* ± *SD* (*n* = 3), ∗*p* < 0.05. IFN: interferon; IL: interleukin; STAT: signal transducer and activator of transcription.

**Figure 9:** Effect of DC-conditioned medium on cytokine production and mRNA expression in Th9 cells. Th9 cells were cultured with conditioned medium was collected from unstimulated or IFN-*γ*-stimulated DCs. (a) ELISA of IFN-*γ,* IL-27, and IL-9 in Th9 cells cultured with or without DC-conditioned medium. (b) qRT-PCR of expression of *IL-9* and *T-bet* mRNA in Th9 cells cultured with or without DC-conditioned medium. Results are presented as *mean* ± *SD* (*n* = 3), ∗*p* < 0.05. IFN: interferon; IL: interleukin; DCs: dendritic cells.

**Figure 10:** Effect of DC-conditioned medium on STAT signaling in Th9 cells. Th9 cells were cultured with conditioned medium collected from unstimulated or IFN-*γ*-stimulated DCs. (a) Western blot of expression of p-STAT1, STAT1, p-STAT3, and STAT3 proteins in Th9 cultured with or without DC-conditioned medium for 20, 60, or 120 min. Quantification of phosphorylation levels of (b) STAT1 and (c) STAT3 relative to respective total protein content. Results are presented as *mean* ± *SD* (*n* = 3), ∗*p* < 0.05; #*p* < 0.05 compared with the same group at 20 min; Δ*p* < 0.05 compared with the same group at 60 min. IFN: interferon; DCs: dendritic cells; STAT: signal transducer and activator of transcription.

**Figure 11:** Proposed mechanism of IFN-*γ*-mediated Th9 differentiation through IL-27 release from DCs. When DCs are stimulated by IFN-*γ*, IL-17 is released, which in turn inhibits the differentiation of CD4+ T cells into a Th9 phenotype and alleviates AA.

**Table 1:** Primer sequences for qRT-PCR.

Primer	Sequence (5′-3′)
IFN-*γ* forward	TAGATGTGGAAGAAAAGA
IFN-*γ* reverse	TTGCTGAAGAAGGTAGTA
IL-27 forward	GCCAGGTGACAGGAGA
IL-27 reverse	GAAACATTGGGAAGAT
IL-27R forward	AAACTTCTGGCAAACG
IL-27R reverse	CAGCACGGGACCTCTT
IL-9 forward	ATCCACCGTCAAAATG
IL-9 reverse	GGAAAACAGGCAAGAG
T-bet forward	TCCCATTCCTGTCCTTCA
T-bet reverse	TGCCTTCTGCCTTTCCAC
*β*-actin forward	CCCATCTACGAGGGCTAT
*β*-actin reverse	TGTCACGCACGATTTCC

**Table 2:** Antibodies for western blot.

Antibody	Host	Supplier	Product code	Dilution	Molecular weight (kDa)
IFN-*γ*	Rabbit	Bioswamp	PAB36509	1:1000	24
*β*-actin	Rabbit	Bioswamp	PAB36265	1:10000	42
p-STAT1	Rabbit	Bioswamp	PAB43467-P	1:1000	87
STAT1	Rabbit	Bioswamp	PAB36419	1:1000	90
p-STAT3	Rabbit	Bioswamp	PAB36302-P	1:1000	88
STAT3	Rabbit	Bioswamp	PAB37351	1:1000	105
Goat anti-rabbit IgG	Goat	Bioswamp	SAB43711	1:10000	

## Data Availability

All data generated or analyzed during this study are included either in this article or in the supplementary information files.
